# A Selection of Trauma Scores Might Not Correlate with Coagulation Factor Activity following Multiple Injuries: A Retrospective Observational Study from a Level 1 Trauma Center

**DOI:** 10.1155/2020/6726017

**Published:** 2020-12-30

**Authors:** Manuel Burggraf, Christina Polan, Heinz-Lothar Meyer, Roman Maximilian Müller, Felix Reinecke, Marcel Dudda, Max Daniel Kauther

**Affiliations:** Department of Trauma, Hand and Reconstructive Surgery, University Hospital Essen, University of Duisburg-Essen, Hufelandstr. 55, Essen 45147, Germany

## Abstract

Loss and dilution of coagulation factors have been observed following multiple trauma. Timely recognition of reduced clotting factor activity might facilitate therapeutic action to restore normal coagulation function. This study investigates the potential role of some well-known trauma scores in predicting coagulation factor activity after multiple injuries. A dataset comprising the coagulation factor activities of 68 multiply injured adult patients was analyzed. The following trauma scores were evaluated: AIS, ISS, NISS, GCS, RTS, TRISS, RISC, and TASH score. To investigate the effect of trauma severity with respect to a single anatomic injury location, two groups according to the AIS (<3 vs. ≥3 points) were formed. Differences between these two groups were analyzed for five different body regions (head, thorax, abdomen, pelvis, extremities) using the Mann–Whitney *U*-test. Spearman's rank correlation coefficient rho was calculated to reveal possible relationships between trauma scores and clotting factor activities. The analysis showed clearly reduced clotting factor activities with a significant reduction of FII (83 *vs.* 50%; *P* = .021) and FV (83 *vs.* 46%; *P* = .008) for relevant (AIS ≥ 3 points) pelvic injuries. In contrast, traumatic brain injury according to the AIS head or the GCS does not appear to lead to a significant decrease in coagulation factor activities. Furthermore, the other scores studied show at best a fair correlation with coagulation factor activity. In this context, the RTS score seems to be the most suitable. Additionally, the predictive value of the TASH score, which was specifically developed to predict the need for mass transfusion, was also limited in this study. We would like to explicitly point out that this is not a criticism of the trauma scores, since they were developed in a completely different context.

## 1. Introduction

Severe trauma is the primary reason for mortality in the younger population worldwide [1]. In many trauma victims, severe bleeding and coagulopathy play a crucial role for lethality [2]. The coagulopathy following trauma is a multifactorial condition which is, among many other factors, partly due to the loss or dilution of coagulation factors [3]. Several studies have demonstrated this loss of coagulation factor activity in various trauma populations [4–9]. Furthermore, it has been shown that mortality is dependent on clotting factor depletion and that different phenotypes of clotting factor alterations are of importance [10, 11]. Unfortunately, the usual coagulation tests such as the International Normalized Ratio (INR) and Partial Thromboplastin Time (PTT) at best only partially reflect the changes at the level of the coagulation factors [4, 5, 12]. Moreover, their results are only available at a relatively late time after injury and point-of-care test systems have proven to be prone to errors [13]. Therefore, a reliable estimate of clotting factor profiles based on easily available clinical findings might be beneficial for the treatment of traumatized patients. Trauma scores have long been used to derive recommendations for action and/or prognoses for seriously injured patients [14]. Besides anatomical injury scores like the well-known Injury Severity Score (ISS), which itself is based on the so-called Abbreviated Injury Scale (AIS), there are also a number of physiological and combined scoring systems [15]. In a recent systematic review, Shih et al. assessed clinical scores and tools to predict the need for activation of a massive transfusion protocol [16]. Nevertheless, to the best of our knowledge, the capability of trauma scores to directly predict changes of clotting factor activities following severe trauma has not been investigated yet. Therefore, the aim of this study was to elucidate the capability of a range of different existing trauma scores in predicting clotting factor activities in the early phase following multiple trauma.

## 2. Materials and Methods

The study is based on an existing dataset of clotting factor activities from multiply injured patients at our institution (level 1 trauma center in Germany) that was published previously [4]. The method description partly reproduces the wording of that study. In brief, blood samples were collected from 68 multiply injured adult patients who met the highest-level trauma activation criteria and who were directly transferred from the scene of the accident to our trauma resuscitation room. Pregnant women and patients with any form of preexisting coagulation alteration including anticoagulants were excluded from the study. The mean age of the patients was 45 ± 17 years, 56 (82%) were male, and the mean ISS was 24 ± 13 points. 13 (19%) patients died with a median survival of 4.9 days (78–30128 minutes). Of these 13 deceased patients, 8 had an AIS head or an AIS thorax ≥ 3 points, 3 had an AIS extremities ≥ 3 points, and one each had an AIS abdomen or AIS pelvis ≥ 3 points. The death rate for relevant injuries (AIS ≥ 3 points) was 35% (AIS head), 25% (AIS abdomen), 21% (AIS thorax and AIS extremities), and 20% (AIS pelvis), respectively. Although the ultimate cause of death is difficult to determine, 10 out of these 13 patients had a documented diagnosis of anemia, and 7 were coagulopathic. Besides standard blood tests, the soluble clotting factors (FII, V, VII, VIII, IX, X, XI, XII, XIII, fibrinogen, and calcium) were analyzed. Their mean activity or level is given together with the INR and PTT in Table 1. For this retrospective observational study, additional clinical data was collected to allow for the evaluation of specific trauma scores. The scores comprise the AIS [17], the ISS [18], the New Injury Severity Score (NISS) [19], the Glasgow Coma Scale (GCS) [20], the Revised Trauma Score (RTS) [21], the Trauma Injury Severity Score (TRISS) [22], the Revised Injury Severity Classification (RISC) [23], and the Trauma Associated Severe Hemorrhage (TASH) score [24]. Whereas the AIS, ISS, NISS, and GCS were known for all patients, the computation of the other scores was possible in only 60 (RISC), 57 (TASH), 46 (RTS), and 45 (TRISS) cases, respectively, due to missing data. The mean values of the scores together with the standard deviation are given in Table 2. The study was carried out in compliance with the Helsinki Declaration and was approved by the relevant local ethics committee (reference 12-5120-BO). Written informed consent was obtained from the participants subsequently after recovery, or in case of permanent impairment or death, the relatives or legal representative were asked for their consent.

IBM® SPSS® Statistics (version 25) was used for statistical analysis. To investigate the effect of trauma severity with respect to a single anatomic injury location, two groups according to the AIS (<3 vs. ≥3 points) were formed. Differences between these two groups were analyzed for five different body regions (head, thorax, abdomen, pelvis, extremities) using the Mann–Whitney *U* test. In this context, the assignment with regard to body region was not based on the complex structure given by the AIS, but on the actual anatomical region of injury. The results are reported as median values with 25 and 75 percentiles. Secondly, potential relationships between the clotting factor activities and several trauma scores were investigated. In order to better assess the results, the analysis was extended to include, besides the aforementioned clotting factors, routine coagulation tests (INR and PTT), levels of hemoglobin and lactate, and transfused units of Packed Red Blood Cells (PRBC) and Fresh Frozen Plasma (FFP). As linear relationship could not be assumed, Spearman's rank correlation coefficient rho (*ρ*) was calculated to reveal possible relationships. Additionally, the 95% confidence interval (CI) was computed by bootstrapping using a bias-corrected and accelerated method based on 1000 bootstrap samples. As proposed by Chan, the strength of correlation was considered poor for absolute values of *ρ* below 0.30, fair between 0.30 and 0.59, moderate between 0.60 and 0.79, and very strong above 0.80 [25]. A *P* value smaller than 0.05 (2-tailed) was considered statistically significant for all tests. All authors had access to primary clinical data.

## 3. Results

Clotting factor profiles for the five specific regions and according to the assessment of injury severity based on the AIS values are shown in Table 3. The analysis showed a significant reduction of FV activity for relevant (AIS ≥ 3 points) thoracic (90 *vs.* 76%; *P* = .031) and pelvic (83 *vs.* 46%; *P* = .008) injuries. Furthermore, relevant pelvic injuries led to a significantly reduced activity of FII (83 *vs.* 50%; *P* = .021). Additionally, the need for PRBC transfusion was significantly higher for patients with relevant pelvic trauma (0 *vs.* 3 units; *P* = .007) or injuries of the extremities (0 *vs.* 2 units; *P* = .005). No further significant differences were found between the groups with low and high AIS values. However, although without consistent significance, a comprehensive decrease of coagulation factor activities was shown for the AIS pelvis ≥ 3 subgroup in contrast to all other regions.

Evaluation of correlation between anatomical trauma scores and clotting factor activities showed a significant fair relationship for the ISS with six (fibrinogen, calcium, FVIII, FIX, FXI, FXII) and for the NISS with four (fibrinogen, calcium, FIX, FXIII) of the eleven clotting factors (Table 4). Whereas both scores demonstrated a fair relationship with hemoglobin, the NISS also showed a fair relationship with PTT and the administration of PRBC. In contrast, none of these tests showed a relevant relationship with INR, levels of lactate, or administered units of FFP.

Table 5 shows the results of the correlation analysis for the physiological trauma scores. The RTS showed significant fair correlations with as many as nine of the coagulation factors (fibrinogen, calcium, FII, FVIII, FIX, FX, FXI, FXII, FXIII), whereas for the GCS this was the case for only one factor (calcium). The physiological scores also had a fair relationship with PTT and levels of hemoglobin and, additionally in the case of the RTS, with INR. Levels of lactate or the need for transfusion were not correlated with either test.

Regarding the combined trauma scores given in Table 6, TRISS showed a significant fair relationship with four clotting factors (fibrinogen, calcium, FII, FXIII), the RISC with just one (FXIII). Additionally, there was a fair relationship between both scores and PTT, whereas only the TRISS also fairly correlated with INR. In contrast, only the RISC had fair correlation with levels of hemoglobin. Neither of the scores showed a relevant relationship with lactate levels or the transfusion of blood products.

Finally, Table 7 shows that the TASH has a significant, moderately strong correlation with levels of calcium and a significant fair correlation to three other clotting factors (fibrinogen, FII, FV). Additionally, there was a fair correlation between the TASH and the INR, levels of hemoglobin, and administration of PRBC and FFP.

## 4. Discussion

To the best of our knowledge, this is the first study to examine the role of some well-known trauma scores as predictors of clotting factor deficiencies following multiple injuries. Our results show that these commonly used scoring systems show at best a fair correlation with the activities or levels of some of the soluble coagulation factors after trauma. We would like to explicitly point out that this is not a criticism of the trauma scores, since they were developed in a completely different context [15].

Historically, the ordinally scaled AIS is not an actual trauma score but was developed to estimate the isolated death probability of specific injuries after traffic accidents, with one point referring to minor and up to six points for currently not survivable injuries. Nowadays, the AIS is also considered a valid marker of the severity of an injury [26]. The results of this study imply that severe pelvic injuries rather than injuries at other anatomic regions are associated with lower activities or levels of coagulation factors, predominantly FII and FV. Patients suffering from these pelvic injuries also had a significantly higher rate of PRBC transfusions. This is in line with recently published data, showing that with increasing injury severity according to the Arbeitsgemeinschaft für Osteosynthese (AO) classification, the rate of blood transfusions within the first six hours after pelvic trauma increases significantly [27]. Our results suppose that severe pelvic injuries are an especially significant cause of trauma-induced coagulopathy at the level of coagulation factor activities and levels. Overall, early and aggressive hemostatic therapy, as suggested by some authors for this patient collective, seems appropriate [28].

As regards the correlation analyses, the anatomic trauma scores ISS and NISS both demonstrated some fair relationships with clotting factor activities. Whereas the ISS is calculated by adding the squared AIS values of the three most severely injured body regions, the NISS is the sum of the squares of the top three AIS scores irrespective of body region [18, 19]. Balogh et al. comparatively assessed both scores, and the NISS seemed to be a better predictor of mortality and complications such as multiple organ failure (MOF) as well as transfusion requirements [29]. We therefore speculated that this might also apply to the prediction of changes in coagulation factor activities. However, this turned out not to be the case. This might be because the calculation of the NISS (in contrast to the ISS) often includes multiple injuries in the extremities, resulting in higher values. But our analysis of the AIS values for the extremities revealed that, with the exception of FXIII, serious injuries in this body region did not lead to significantly reduced levels of coagulation factor activity (Table 3). Additionally, although only the NISS showed a fair correlation with the administration of PRBC, the absolute difference to the ISS with respect to rho is minimal (Table 4). Therefore, the potential clinical relevance is probably very low. Husum and Strada, comparing the ISS and NISS for penetrating injuries, argued that the superiority of the NISS over the ISS was lower in terms of predicting complications and MOF than in terms of mortality [30]. Furthermore, according to Husum et al., the predictive accuracy of the ISS and NISS for postinjury complications and MOF may be regarded as only “fair,” which in principle is in line with the findings of this study for clotting factor activities and levels.

Of the four physiological or combined trauma scores, the GCS must be considered separately, as it only evaluates cerebral function [20]. Coagulation disorders associated with traumatic brain injury (TBI) have been known for a long time, but what exactly triggers their development is still not fully understood [31]. Indeed, it has been shown that lower GCS values are related to coagulopathy in injured adults and children alike [32]. Yet, the GCS in our study was only a poor indicator of coagulation factor activity (Table 5). Nevertheless, this is in line with the findings of Cohen et al., who showed that TBI only leads to early coagulopathy in conjunction with hypoperfusion and that this coagulopathy is not due to consumption of clotting factors [33]. This is further supported by our results which show that even a relevant TBI according to the AIS did not lead to a significant reduction of coagulation factor activity (Table 3). In this context, it must be pointed out that the patient collective we examined in this study was a heterogeneous group of severely injured and not an isolated TBI cohort. The potential effects of craniocerebral trauma could therefore have been overlaid by other relevant accompanying injuries. Interestingly, the RTS, which is calculated using a complex formula based on the GCS, systolic blood pressure, and breathing rate [21], showed the most extensive correlations with coagulation factor activity (Table 5). Ultimately, this underlines the statements made above, as the addition of physiologic indicators of hypoperfusion to the GCS substantially enhanced the range of at least fair correlations of the RTS with clotting factors. However, the RTS did not correlate with the amount of PRBC or FFP administered. Furthermore, an important limitation is that the RTS can only be formally calculated for patients still breathing spontaneously in the resuscitation room. Alternatively, the breathing rate prior to intubation at the accident site can be used [15]. Since this information is notoriously lacking, in the end, only the data of 46 patients could be analyzed in our collective. Therefore, a selection bias cannot be excluded with certainty.

Again, it was shown that hypoperfusion generally leads to reduced coagulation factor activity [8]. We had therefore suspected in advance that scoring systems incorporating shock markers should have been superior in predicting clotting factor deficiencies. Whereas the RTS, at least to some extent, confirmed this, the TRISS and especially the RISC showed only a few correlations of fair extent (Table 6). Like the RTS, both scores use complex algorithms and were developed to predict the survival probabilities of multiply injured patients [22, 23]. The calculation of the TRISS requires the ISS, the RTS, the patient age, and the trauma mechanism (blunt *vs.* penetrating). The same limitations with respect to data availability apply as for the RTS itself, so that ultimately only 45 patients could be included. Overall, we assume that the low correlation of the TRISS with some of the coagulation factors is probably mainly due to the incorporation of the RTS. This limited predictive power of the TRISS in terms of coagulation factor activity is in line with the finding that the TRISS also underestimates mortality in the presence of a coagulation disorder [34]. With regard to the RISC, this score was developed and validated with data from the Trauma Registry of the German Society for Trauma Surgery [23]. Several variables are included in its calculation (age, NISS, AIS head and extremities, GCS, PTT, base excess, resuscitation, indirect bleeding signs). In view of these parameters, correlations with coagulation factor activity could have been expected, yet none were found. All in all, the principally observed limitation of the latter three scores with regard to the objective of this study probably lay in the fundamental fact that they use mathematical weighting factors for the clinical variables used, which were specifically developed and validated to predict mortality, not coagulopathy in any form [15].

In this context, we also analyzed a score which was specifically developed and validated to predict the probability of mass transfusion after multiple trauma [24, 35]. The TASH score is based on a logistic function of several clinical markers (sex, hemoglobin, base excess, systolic blood pressure, heart rate, injuries, or findings suspected of bleeding). From the various existing scores predicting massive transfusion after multiple injuries, we chose the TASH score because this score is well validated, and its overall accuracy seems to be superior to others [16, 36, 37]. Indeed, of all the scores in our study the TASH score showed the best, although only fair, correlation with the number of PRBC and FFP transfusions. Hence, in terms of coagulation factor activity, the correlation in general was neither comprehensive nor particularly pronounced (Table 7). It should be noted, however, that the TASH score was not designed to indicate the need for transfusion in general, but for the necessity of a mass transfusion (≥10 units of PRBC). Overall, the transfusion rate of PRBC in this study was 26%, whereas the massive transfusion rate was only 3%. Sensitivity to minor derangements, therefore, could be limited due to the focus on massive transfusion in the development of this score. However, it has been shown in another study that the TASH score does correlate with lower numbers of PRBC as well [37].

## 5. Limitations

Some general limitations apply to this study. First of all, it is of retrospective observational character and therefore prone to various known types of bias [38]. Secondly, it is based on a rather small number of patients. Therefore, possible correlations could have remained undiscovered. Furthermore, analysis of clotting factor activities according to specific AIS values and regions, respectively, might be biased, as these groups do not represent isolated injuries. An influence by relevant concomitant injuries can therefore not be excluded with conclusive certainty. Additionally, patient characteristics in terms of trauma mechanism differ considerably between the various studies mentioned above. For instance, whereas the study of Husum et al. solely investigated penetrating injuries, the rate of penetrating injuries in this study was only 4% [4, 30]. However, with the exception of FXIII, our previous study showed no significant differences in coagulation factor activity between patients with blunt or penetrating trauma [4]. Furthermore, the analysis of the correlation between the different scores and transfusion requirements depends at least partially on how liberal or restrictive PRBC and/or FFP are transfused. Therefore, it cannot be ruled out that these results are subject to variations according to the transfusion protocols of single institutions. Finally, since this is not an interventional study, no valid statements can be made about potential therapeutic changes derived from its findings.

### 5.1. Future Directions

Over the last decade, two major strategies for coagulation management have evolved. On the one hand, the implementation of massive transfusion protocols, based on the application of a fixed ratio of blood products (with a considerable variance between the individual institutions), led to a reduction of mortality in trauma patients [39]. On the other hand, the introduction of viscoelastic tests to guide “individualized” resuscitation therapy showed promising results with regard to the use of blood products and overall mortality [40]. In the future, the identification of the ideal resuscitation product will increasingly come into focus [41]. We are convinced that knowledge of the changes in the individual coagulation factors is of great importance for this purpose. Yet, there is a paucity on studies linking coagulation factor activities to easily available clinical data. Despite the limitations described above, this study reveals some interesting new aspects that indicate further investigation. Although none of the trauma scores examined could show a superior correlation with coagulation factor activity in general, there was evidence that the use of certain physiological parameters may be appropriate to indicate changes in coagulation factor activity. In addition, the effects of different trauma entities (e.g., TBI versus pelvis) on coagulation factors should be investigated in larger clinical studies. The overall goal should be to develop the best possible empirical coagulation therapy in the early posttrauma phase.

## 6. Conclusions

The values of some common trauma scores are only poorly correlated with coagulation factor activity. The results of our study show that the RTS score seems to be the most suitable in this respect. Unfortunately, the predictive value of the TASH score, which was specifically developed to predict the need for mass transfusion, is also limited regarding the objectives of this study. Importantly, none of the scores was explicitly developed to make a statement about the specific condition of clotting factor deficiencies, and testing them in this regard is obviously somewhat unfair. We therefore explicitly do not want our statements to be understood as a criticism of the scores. Although, as discussed above, a certain bias by concomitant injuries cannot be fully excluded, severe pelvic injuries rather than TBI seem to be related to reduced clotting factor activities and higher transfusion rates of PRBC. Overall, reliable but also easily available indicators for the loss or consumption of clotting factors as a specific cause of coagulopathy after severe multiple trauma are still urgently needed.

## Figures and Tables

**Table 1:** Activities or levels of soluble clotting factors, INR, and PTT from 68 multiply injured patients.

	Mean	SD
Fibrinogen (mg/dl)	244	74
FII (%)	82	20
Calcium (mmol/l)	2.12	0.15
FV (%)	79	22
FVII (%)	89	23
FVIII (%)	216	90
FIX (%)	97	25
FX (%)	87	23
FXI (%)	101	26
FXII (%)	94	33
FXIII (%)	92	28
INR	1.09	0.14
PTT (sec)	26.7	6.5

Standard deviation (SD), clotting factor (F), International Normalized Ratio (INR), Partial Thromboplastin Time (PTT).

**Table 2:** Mean values with a standard deviation of the different scores.

Points	Mean	SD	*n*
ISS	24	13	68
NISS	31	19	68
GCS	11	5	68
RTS	6.372	2.086	46
TRISS	76.3	33.2	45
RISC	83.3	25.9	60
TASH	5	4	57

Standard deviation (SD), Injury Severity Score (ISS), New Injury Severity Score (NISS), Glasgow Coma Scale (GCS), Revised Trauma Score (RTS), Trauma Injury Severity Score (TRISS), Revised Injury Severity Classification (RISC), Trauma Associated Severe Hemorrhage (TASH) score.

**Table 3:** Comparison of clotting factor activities and levels for different regions according to the AIS.

	Head			Thorax			Abdomen			Pelvis			Extremities		
	AIS<3 (*n* = 45)	AIS ≥3 (*n* = 23)	*P*	AIS < 3 (*n* = 29)	AIS ≥ 3 (*n* = 39)	*P*	AIS < 3 (*n* = 64)	AIS ≥ 3 (*n* = 4)	*P*	AIS < 3 (*n* = 63)	AIS ≥ 3 (*n* = 5)	*P*	AIS < 3 (*n* = 54)	AIS ≥ 3 (*n* = 14**)**	*P*
Fibrinogen (mg/dl)	237 (212-296)	235 (206-268)	.418	237 (213-280)	237 (210-273)	.995	237 (210-275)	228 (134-367)	.754	237 (210-275)	230 (152-268)	.452	237 (216-284)	227 (156-267)	.228
FII (%)	84 (71-97)	73 (65-91)	.201	87 (71-106)	80 (67-92)	.104	81 (68-95)	85 (74-88)	.927	**83 (71-95)**	**50 (44-80)**	**.021** ^∗^	84 (69-95)	79 (62-96)	.430
Calcium (mmol/l)	2.16 (2.10-2.23)	2.10 (1.96-2.20)	.163	2.16 (1.97-2.25)	2.10 (2.06-2.20)	.582	2.14 (2.06-2.22)	1.93 (1.88-2.14)	.086	2.12 (2.05-2.20)	2.28 (2.07-2.30)	.154	2.14 (2.06-2.20)	2.10 (1.85-2.22)	.193
FV (%)	80 (71-97)	78 (53-90)	.152	**90 (70-98)**	**76 (56-88)**	**.031** ^∗^	80 (66-96)	77 (68-89)	.658	**83 (69-96)**	**46 (37-73)**	**.008** ^∗∗^	80 (67-91)	85 (53-97)	.756
FVII (%)	89 (66-103)	90 (79-100)	.418	90 (74-100)	90 (70-105)	.724	90 (71-102)	91 (64-100)	.735	90 (73-102)	64 (63-92)	.110	90 (73-102)	89 (64-100)	.462
FVIII (%)	231 (138-309)	184 (138-265)	.504	208 (127-317)	207 (140-261)	.780	204 (137-277)	245 (180-325)	.376	208 (136-278)	168 (139-277)	.796	196 (137-268)	258 (135-306)	.363
FIX (%)	95 (81-119)	89 (80-110)	.351	94 (84-120)	94 (77-108)	.379	94 (80-112)	99 (90-120)	.523	94 (82-112)	74 (67-113)	.301	93 (80-113)	97 (79-111)	.739
FX (%)	88 (73-102)	87 (69-94)	.560	90 (73-100)	86 (70-101)	.577	87 (70-100)	90 (75-98)	.764	88 (75-101)	58 (47-91)	.063	89 (70-101)	87 (69-98)	.481
FXI (%)	99 (88-114)	99 (85-117)	.826	106 (88-121)	97 (88-111)	.564	99 (87-116)	99 (88-124)	.938	99 (88-117)	91 (68-118)	.481	99 (88-117)	101 (82-117)	.856
FXII (%)	91 (77-109)	94 (70-112)	.974	91 (70-113)	91 (75-108)	.547	93 (76-111)	80 (62-91)	.216	91 (75-109)	85 (45-116)	.424	91 (77-109)	93 (52-117)	.820
FXIII (%)	88 (73-114)	83 (68-108)	.273	83 (65-115)	89 (76-112)	.217	88 (73-112)	58 (50-102)	.076	87 (73-112)	65 (54-119)	.277	88 (73-113)	79 (62-91)	.141
INR	1.05 (0.99-1.13)	1.08 (1.03-1.18)	.161	1.04 (1.00-1.10)	1.08 (1.01-1.14)	.286	1.06 (1.00-1.13)	1.05 (1.00-1.17)	.938	1.05 (1.00-1.12)	1.13 (1.08-1.25)	.080	1.06 (1.01-1.11)	1.10 (1.00-1.25)	.395
PTT (sec)	24.8 (23.2-27.4)	27.4 (23.5-29.9)	.101	25.3 (23.2-27.8)	25.4 (23.4-28.8)	.598	25.3 (23.3-28.5)	25.7 (23.0-27.6)	.948	25.3 (23.2-28.0)	29.3 (24.0-31.1)	.254	25.4 (23.4-28.0)	24.4 (22.6-29.9)	.808
Hemoglobin (g/dl)	13.0 (11.3-14.2)	12.2 (11.1-13.4)	.175	12.9 (11.2-14.2)	12.8 (11.1-13.9)	.701	13.0 (11.4-14.1)	10.9 (8.9-12.5)	.072	13.0 (11.4-14.0)	11.1 (10.1-13.9)	.397	13.0 (11.4-14.0)	12.1 (9.1-14.0)	.413
PRBC (*n*)	0 (0-1)	0 (0-2)	.880	0 (0-0)	0 (0-3)	.358	0 (0-2)	0 (0-35)	.827	**0 (0-0)**	**3 (1-7)**	**.007** ^∗∗^	**0 (0-0)**	**2 (0-5)**	**.005** ^∗∗^
FFP (*n*)	0 (0-0)	0 (0-0)	.258	0 (0-0)	0 (0-0)	.944	0 (0-0)	0 (0-41)	.256	0 (0-0)	0 (0-3)	.518	0 (0-0)	0 (0-2)	.117

AIS: Abbreviated Injury Scale; F: clotting factor; INR: International Normalized Ratio; PTT: Partial Thromboplastin Time; PRBC: Packed Red Blood Cells; FFP: Fresh Frozen Plasma. ^∗^*P* < .05; ^∗∗^*P* < .01; Mann–Whitney-U-Test with median values (25-75 percentiles). Significant results were marked in bold.

**Table 4:** Correlation of anatomical trauma scores with clotting factor activities or levels and clinical data.

Spearman's rho	ISS *n* = 68				NISS *n* = 68			
	*r*	95% CI		*P*	*r*	95% CI		*P*
		Lower	Upper			Lower	Upper	
Fibrinogen	**-.36**	**-.60**	**-.05**	**.024**	**-.35**	**-.56**	**-.10**	**.007**
FII	-.27	-.55	.10	.092	-.23	-.45	.02	.080
Calcium	**-.32**	**-.59**	**.02**	**.045**	**-.35**	**-.58**	**-.10**	**.007**
FV	-.14	-.50	.24	.386	-.23	-.46	.02	.077
FVII	-.03	-.33	.27	.847	-.04	-.31	.22	.785
FVIII	**-.34**	**-.64**	**.03**	**.031**	-.10	-.36	.18	.447
FIX	**-.48**	**-.75**	**-.12**	**.002**	**-.30**	**-.53**	**-.06**	**.020**
FX	-.18	-.48	.17	.270	-.21	-.45	.05	.110
FXI	**-.48**	**-.73**	**-.11**	**.002**	-.26	-.49	.00	.047
FXII	**-.33**	**-.61**	**.03**	**.038**	-.23	-.47	.02	.085
FXIII	-.26	-.56	.06	.103	**-.30**	**-.52**	**-.04**	**.022**
INR	.22	-.02	.43	.081	.27	.02	.48	.040
PTT	.27	.02	.50	.028	**.31**	**.06**	**.53**	**.018**
Hemoglobin	**-.31**	**-.56**	**.00**	**.012**	**-.35**	**-.54**	**-.12**	**.008**
Lactate	.15	-.10	.39	.239	.15	-.18	.44	.270
PRBC	.28	.01	.51	.024	**.31**	**.06**	**.51**	**.020**
FFP	.07	-.16	.30	.605	.17	-.15	.42	.201

ISS: Injury Severity Score; NISS: New Injury Severity Score; CI: confidence interval; F: clotting factor; INR: International Normalized Ratio; PTT: Partial Thromboplastin Time; PRBC: Packed Red Blood Cells; FFP: Fresh Frozen Plasma. Results of ISS partially reproduced from [4]. Significant results of at least fair relationship were marked in bold.

**Table 5:** Correlation of physiological trauma scores with clotting factor activities or levels and clinical data.

Spearman's rho	GCS *n* = 68				RTS *n* = 46			
	*r*	95% CI		*P*	*r*	95% CI		*P*
		Lower	Upper			Lower	Upper	
Fibrinogen	.27	.03	.49	.029	**.44**	**.18**	**.63**	**.003**
FII	.16	-.08	.38	.206	**.49**	**.27**	**.68**	**.001**
Calcium	**.36**	**.09**	**.57**	**.004**	**.59**	**.33**	**.77**	**.000**
FV	.17	-.08	.39	.185	.30	-.01	.54	.053
FVII	-.07	-.30	.18	.599	.20	-.10	.46	.208
FVIII	.18	-.04	.38	.149	**.32**	**.04**	**.59**	**.036**
FIX	.16	-.08	.38	.198	**.41**	**.13**	**.63**	**.008**
FX	.13	-.10	.36	.313	**.37**	**.10**	**.62**	**.015**
FXI	.11	-.12	.33	.394	**.40**	**.12**	**.64**	**.008**
FXII	.14	-.14	.37	.262	**.50**	**.25**	**.69**	**.001**
FXIII	.29	.04	.52	.018	**.54**	**.30**	**.71**	**.000**
INR	-.19	-.44	.06	.143	**-.41**	**-.65**	**-.07**	**.008**
PTT	**-.34**	**-.56**	**-.05**	**.006**	**-.47**	**-.76**	**-.11**	**.002**
Hemoglobin	**.33**	**.08**	**.55**	**.009**	**.51**	**.25**	**.72**	**.001**
Lactate	-.21	-.45	.04	.090	-.30	-.57	.04	.056
PRBC	.08	-.23	.40	.551	-.17	-.48	.17	.268
FFP	.17	-.18	.38	.190	-.06	-.44	.25	.683

GCS: Glasgow Coma Scale; RTS: Revised Trauma Score; CI: confidence interval; F: clotting factor; INR: International Normalized Ratio; PTT: Partial Thromboplastin Time; PRBC: Packed Red Blood Cells; FFP: Fresh Frozen Plasma. Significant results of at least fair relationship were marked in bold.

**Table 6:** Correlation of combined trauma scores with clotting factor activities or levels and clinical data.

Spearman's rho	TRISS *n* = 45				RISC *n* = 60			
	*r*	95% CI		*P*	*r*	95% CI		*P*
		Lower	Upper			Lower	Upper	
Fibrinogen	**.36**	**.07**	**.59**	**.019**	.21	-.08	.47	.127
FII	**.40**	**.08**	**.66**	**.010**	.24	-.02	.47	.078
Calcium	**.40**	**.12**	**.62**	**.009**	.26	-.04	.52	.056
FV	.22	-.11	.51	.167	.10	-.19	.35	.464
FVII	.09	-.24	.42	.589	.09	-.21	.39	.512
FVIII	.25	-.08	.56	.120	.12	-.14	.38	.381
FIX	.26	-.12	.60	.105	.14	-.17	.45	.294
FX	.25	-.09	.56	.119	.19	-.08	.44	.172
FXI	.30	-.06	.63	.053	.20	-.09	.50	.149
FXII	.28	-.07	.61	.073	.12	-.14	.38	.387
FXIII	**.49**	**.22**	**.69**	**.001**	**.35**	**.09**	**.57**	**.008**
INR	**-.37**	**-.64**	**-.08**	**.016**	-.23	-.45	-.01	.086
PTT	**-.52**	**-.73**	**-.26**	**.000**	**-.35**	**-.57**	**-.12**	**.008**
Hemoglobin	.27	-.01	.53	.086	**.31**	**.05**	**.52**	**.022**
Lactate	-.23	-.53	.10	.147	-.21	-.49	.10	.121
PRBC	-.11	-.38	.14	.480	-.21	-.45	.04	.115
FFP	-.03	-.31	.20	.830	-.13	-.34	.14	.336

TRISS: Trauma Score–Injury Severity Score; RISC: Revised Injury Severity Classification; CI: confidence interval; F: clotting factor; INR: International Normalized Ratio; PTT: Partial Thromboplastin Time; PRBC: Packed Red Blood Cells; FFP: Fresh Frozen Plasma. Significant results of at least fair relationship were marked in bold.

**Table 7:** Correlation of the Trauma Associated Severe Hemorrhage (TASH) score with clotting factor activities or levels and clinical data.

Spearman's rho	TASH *n* = 57			
	*r*	95% CI		*P*
		Lower	Upper	
Fibrinogen	**-.34**	**-.59**	**-.06**	**.012**
FII	**-.37**	**-.58**	**-.12**	**.007**
Calcium	**-.62**	**-.79**	**-.38**	**.000**
FV	**-.39**	**-.60**	**-.15**	**.004**
FVII	-.21	-.44	.02	.125
FVIII	-.05	-.30	.19	.741
FIX	-.27	-.49	-.03	.054
FX	-.29	-.52	-.03	.036
FXI	-.29	-.52	-.04	.037
FXII	-.20	-.44	.05	.158
FXIII	-.26	-.55	.02	.056
INR	**.36**	**.09**	**.58**	**.009**
PTT	.22	-.07	.49	.117
Hemoglobin	**-.54**	**-.75**	**-.29**	**.000**
Lactate	.29	.05	.51	.032
PRBC	**.43**	**.17**	**.62**	**.001**
FFP	**.43**	**.24**	**.60**	**.001**

TASH score: Trauma Associated Severe Hemorrhage score; CI: confidence interval; F: clotting factor; INR: International Normalized Ratio; PTT: Partial Thromboplastin Time; PRBC: Packed Red Blood Cells; FFP: Fresh Frozen Plasma. Significant results of at least fair relationship were marked in bold.

## References

[1] WHO (2018). *Global Health Estimates 2016: Deaths by Cause, Age, Sex, by Country and by Region, 2000-2016*.

[2] Kauvar D. S., Lefering R., Wade C. E. (2006). Impact of hemorrhage on trauma outcome: an overview of epidemiology, clinical presentations, and therapeutic considerations. *The Journal of Trauma*.

[3] Hess J. R., Brohi K., Dutton R. P. (2008). The coagulopathy of trauma: a review of mechanisms. *The Journal of Trauma*.

[4] Burggraf M., Payas A., Schoeneberg C., Wegner A., Kauther M. D., Lendemans S. (2016). Evaluation of potential clinical surrogate markers of a trauma induced alteration of clotting factor activities. *BioMed Research International*.

[5] Burggraf M., Payas A., Kauther M. D., Schoeneberg C., Lendemans S. (2015). Evaluation of clotting factor activities early after severe multiple trauma and their correlation with coagulation tests and clinical data. *World Journal of Emergency Surgery*.

[6] Cohen M. J., Kutcher M., Redick B. (2013). Clinical and mechanistic drivers of acute traumatic coagulopathy. *Journal of Trauma and Acute Care Surgery*.

[7] Rizoli S. B., Scarpelini S., Callum J. (2011). Clotting factor deficiency in early trauma-associated coagulopathy. *The Journal of Trauma*.

[8] Jansen J. O., Scarpelini S., Pinto R., Tien H. C., Callum J., Rizoli S. B. (2011). Hypoperfusion in severely injured trauma patients is associated with reduced coagulation factor activity. *The Journal of Trauma*.

[9] Burggraf M., Polan C., Husen M. (2020). Trauma induced clotting factor depletion in severely injured children: a single center observational study. *World Journal of Emergency Surgery*.

[10] Kunitake R. C., Howard B. M., Kornblith L. Z. (2017). Individual clotting factor contributions to mortality following trauma. *Journal of Trauma and Acute Care Surgery*.

[11] Kutcher M. E., Ferguson A. R., Cohen M. J. (2013). A principal component analysis of coagulation after trauma. *Journal of Trauma and Acute Care Surgery*.

[12] Stettler G. R., Moore E. E., Moore H. B. (2019). Variability in international normalized ratio and activated partial thromboplastin time after injury are not explained by coagulation factor deficits. *Journal of Trauma and Acute Care Surgery*.

[13] Davenport R., Manson J., De’Ath H. (2011). Functional definition and characterization of acute traumatic coagulopathy. *Critical Care Medicine*.

[14] G Polytrauma Guideline Update (2018). Level 3 guideline on the treatment of patients with severe/multiple injuries: AWMF Register-Nr. 012/019. *European Journal of Trauma and Emergency Surgery*.

[15] Kulla M., Fischer S., Helm M., Lampl L. (2005). Traumascores für den Schockraum - eine kritische Übersicht. *Anästhesiologie, Intensivmedizin, Notfallmedizin, Schmerztherapie*.

[16] Shih A. W., al Khan S., Wang A. Y. (2019). Systematic reviews of scores and predictors to trigger activation of massive transfusion protocols. *Journal of Trauma and Acute Care Surgery*.

[17] Gennarelli T. A., Wodzin E. (2008). *The Abbreviated Injury Scale 2005. Update 2008*.

[18] Baker S. P., O’Neill B. (1976). The injury severity SCORE. *The Journal of Trauma*.

[19] Osler T., Baker S. P., Long W. (1997). A modification of the injury severity score that both improves accuracy and simplifies scoring. *The Journal of Trauma: Injury, Infection, and Critical Care*.

[20] Teasdale G., Jennett B. (1974). Assessment of coma and impaired consciousness. A practical scale. *Lancet*.

[21] Champion H. R., Sacco W. J., Copes W. S., Gann D. S., Gennarelli T. A., Flanagan M. E. (1989). A revision of the trauma score. *The Journal of Trauma*.

[22] Boyd C. R., Tolson M. A., Copes W. S. (1987). Evaluating trauma care. *The Journal of Trauma*.

[23] Lefering R. (2009). Development and validation of the revised injury severity classification score for severely injured patients. *European Journal of Trauma and Emergency Surgery*.

[24] Maegele M., Lefering R., Wafaisade A. (2011). Revalidation and update of the TASH-Score: a scoring system to predict the probability for massive transfusion as a surrogate for life-threatening haemorrhage after severe injury. *Vox Sanguinis*.

[25] Chan Y. H. (2003). Biostatistics 104: correlational analysis. *Singapore Medical Journal*.

[26] Haasper C., Junge M., Ernstberger A. (2010). Die abbreviated injury scale (AIS). *Unfallchirurg*.

[27] Yang Q., Wang T., Ai L. (2020). Clinical outcomes of blood transfusion to patients with pelvic fracture in the initial 6 h from injury. *Experimental and Therapeutic Medicine*.

[28] Joseph B., Khalil M., Harrison C. (2016). Assessing the efficacy of prothrombin complex concentrate in multiply injured patients with high-energy pelvic and extremity fractures. *Journal of Orthopaedic Trauma*.

[29] Balogh Z., Offner P. J., Moore E. E., Biffl W. L. (2000). NISS predicts postinjury multiple organ failure better than the ISS. *The Journal of Trauma: Injury, Infection, and Critical Care*.

[30] Husum H., Strada G. (2002). Injury severity score versus new injury severity score for penetrating injuries. *Prehospital and Disaster Medicine*.

[31] Laroche M., Kutcher M. E., Huang M. C., Cohen M. J., Manley G. T. (2012). Coagulopathy after traumatic brain injury. *Neurosurgery*.

[32] Dwivedi A. K., Sharma A., Sinha V. D. (2018). Comparative study of derangement of coagulation profile between adult and pediatric population in moderate to severe traumatic brain injury: a prospective study in a tertiary care trauma center. *Asian J Neurosurg*.

[33] Cohen M. J., Brohi K., Ganter M. T., Manley G. T., Mackersie R. C., Pittet J. F. (2007). Early coagulopathy after traumatic brain injury: the role of hypoperfusion and the protein C pathway. *The Journal of Trauma: Injury, Infection, and Critical Care*.

[34] Kim S. J., Lee S. W., Han G. S., Moon S. W., Choi S. H., Hong Y. S. (2012). Acute traumatic coagulopathy decreased actual survival rate when compared with predicted survival rate in severe trauma. *Emergency Medicine Journal*.

[35] Y??cel N., Lefering R., Maegele M. (2006). Trauma Associated Severe Hemorrhage (TASH)-Score: probability of mass transfusion as surrogate for life threatening hemorrhage after multiple trauma. *The Journal of Trauma: Injury, Infection, and Critical Care*.

[36] Brockamp T., Nienaber U., Mutschler M. (2012). Predicting on-going hemorrhage and transfusion requirement after severe trauma: a validation of six scoring systems and algorithms on the TraumaRegister DGU. *Critical Care*.

[37] Boutefnouchet T., Gregg R., Tidman J., Isaac J., Doughty H. (2015). Emergency red cells first: rapid response or speed bump? The evolution of a massive transfusion protocol for trauma in a single UK centre. *Injury*.

[38] Hammer G. P., du Prel J. B., Blettner M. (2009). Avoiding bias in observational Studies. *Deutsches Ärzteblatt International*.

[39] Consunji R., Elseed A., El-Menyar A. (2020). The effect of massive transfusion protocol implementation on the survival of trauma patients: a systematic review and meta-analysis. *Blood Transfusion*.

[40] Dhara S., Moore E. E., Yaffe M. B., Moore H. B., Barrett C. D. (2020). Modern management of bleeding, clotting, and coagulopathy in trauma patients: what is the role of viscoelastic assays?. *Curr Trauma Rep*.

[41] Osama M., Syed S. H., Nasir H., Zaidi S. R. (2020). Four-factor prothrombin complex concentrate: an indispensable adjunct in coagulopathy of trauma management - a comparative review of the literature over 2 decades. *European Surgical Research*.

